# Functional Magnetic Resonance Imaging Study of Electroacupuncture Stimulating Uterine Acupoints

**DOI:** 10.1155/2022/4295985

**Published:** 2022-01-19

**Authors:** ChengChao Xu, XiaoHua Yu, Liang Yin, Xiang Li, WanLi Zhang, Fei Li, TianYu Bai

**Affiliations:** ^1^Shandong Provincial Third Hospital, Shandong University, Jinan, Shandong 250031, China; ^2^Shandong University of Traditional Chinese Medicine, Shandong, Jinan 250355, China; ^3^School of Economics, Beijing Technology and Business University, 100048, China

## Abstract

**Objective:**

Based on resting-state functional magnetic resonance imaging (rs-fMRI), to observe the changes of brain function of bilateral uterine points stimulated by electroacupuncture, so as to provide imaging basis for acupuncture in the treatment of gynecological and reproductive diseases.

**Methods:**

20 healthy female subjects were selected to stimulate bilateral uterine points (EX-CA1) by electroacupuncture. FMRI data before and after acupuncture were collected. The ReHo values before and after acupuncture were compared by using the analysis method of regional homogeneity (ReHo) of the whole brain, so as to explore the regulatory effect of acupuncture intervention on brain functional activities of healthy subjects.

**Results:**

Compared with before acupuncture, the ReHo values of the left precuneus lobe, left central posterior gyrus, calcarine, left lingual gyrus, and cerebellum decreased significantly after acupuncture.

**Conclusion:**

Electroacupuncture at bilateral uterine points can induce functional activities in brain areas such as the precuneus, cerebellum, posterior central gyrus, talform sulcus, and lingual gyrus. The neural activities in these brain areas may be related to reproductive hormone level, emotional changes, somatic sensation, and visual information. It can clarify the neural mechanism of acupuncture at uterine points in the treatment of reproductive and gynecological diseases to a certain extent.

## 1. Introduction

Functional magnetic resonance imaging (fMRI) technology is a new noninvasive, nonradioactive, and multiangle method to detect local brain functional activities. FMRI technology has made many achievements in the study of brain functional changes and has been gradually applied to the study of the mechanism of acupuncture and moxibustion in recent years [1, 2]. Uterine acupoint (ex-ca1) is one of the odd acupoints outside the meridian. It has the effects of warming the uterus and regulating menstruation, promoting qi and relieving pain, raising Yang, and lifting depression. It is widely used to treat gynecological diseases such as irregular menstruation, dysmenorrhea, infertility, and uterine prolapse [3]. Because it is located in the less abdomen and is outside the uterus, it is also the main acupoint for regulating the uterus [4]. However, at present, there are few studies on the effective mechanism of uterine acupoints in the treatment of gynecological diseases. Therefore, through functional magnetic resonance imaging technology, we preliminarily explore the effect of electroacupuncture stimulating bilateral uterine acupoints on brain function, so as to provide imaging basis for further exploring the mechanism of acupuncture and moxibustion.

## 2. Materials and Methods

### 2.1. Observation Object

Through the official account of WeChat, the public health volunteers were recruited openly. Inclusion criteria were as follows: (1) age 20-40 years; (2) female, all right-handed; (3) no history of mental or nervous system diseases; (4) menstruation is generally normal; (5) no drug-taking history and acupuncture treatment history within the first two weeks of participating in this project; and (6) those who sign the informed consent form. Exclusion criteria were as follows: (1) those with contraindications to MRI scanning, such as foreign bodies such as metal products, cardiac pacemakers, and metal dentures (which cannot be removed), those with claustrophobia, or those who cannot accept MRI scanning for other reasons; (2) pregnant and lactating women; (3) have a history of alcohol or drug abuse; and ④ those with contraindications to acupuncture and moxibustion. This study was approved by the ethics committee of the Third Hospital of Shandong Province (ethics No.: kyll-2021038). All volunteers were informed of the whole experimental process and signed informed consent.

### 2.2. Electroacupuncture Stimulation Method

Volunteers lie flat on the treatment bed and expose their small abdomen. Huatuo brand disposable acupuncture needle of 0.25∗40 mm is selected as the needle. After routine disinfection of acupoints, the needle is directly inserted into the skin for about 25 mm. After needling qi, connect the Huatuo brand electroacupuncture instrument to both uterine points; select continuous wave, frequency 1 Hz; and keep the needle for 20 min. All 20 volunteers were operated by the same acupuncturist. FMRI scans were performed before and after acupuncture.

### 2.3. MRI Scanning Program and Parameters

The Philips Ingenia 3.0 T MRI scanner of our hospital was used to collect data with 16-channel head neck combined coil, with antinoise earplugs inside and sponge outside. Before examination, the subjects lay flat on the examination bed and had a full rest to eliminate psychological factors such as fear and anxiety. Keep the head still during the examination, wear eye masks, and guide the subjects to relax, not fall asleep, and not do any thinking activities.

Before acupuncture treatment, subjects with intracranial organic lesions were excluded by routine sequence MRI scanning. The scanning sequence included T1WI, T2WI, FLAIR, and DWI. Then, 3D structure data acquisition and finally rs-fMRI (FE-EPI sequence) scanning were done, scanning parameters:TR = 2000 ms,TE = 30 ms,FA = 90°,FOV = 220 mm × 220 mm,matrix = 64 × 64,number of layers = 24,layer thickness = 3 mm,thickness interval = 1 mm; a total of 180 time points were collected. After acupuncture treatment, 3D structural data and RS fMRI were collected.

### 2.4. fMRI Image Processing

In order to reduce the impact of data acquisition error on subsequent analysis results, DPABI software based on MATLAB 2018b platform is used in this project to preprocess the collected MRI data. The preprocessing steps include eliminating the first 10 scanning time points, time horizon correction, and head movement correction (excluding subjects with average head movement amplitude > 1 mm or rotation parameter > 1° in the *X*-, *Y*-, and *Z*-axes). The corrected data will be registered on the EPI template for spatial standardization, and the fMRI image will be resampled with the size of 3 mm × 3 mm × 3 mm voxel. The 24 friston head movement parameters, cerebrospinal fluid, white matter, and whole brain mean signals were removed as covariates. A band-pass filter with a filtering range of 0.01-0.1 Hz was used to eliminate the impact of noise caused by subjects' physiological activities such as breathing and heartbeat on the research results.

### 2.5. Statistical Analysis

After fMRI data preprocessing, DPARSF, SPM8, and other toolkits based on MATLAB platform were used for whole brain regional homogeneity (ReHo) analysis. ReHo analysis can consider local spatial and temporal information at the same time [5]. Kendall concordance coefficient (KCC) can be used to explain the voxel consistency of brain functional regions in different time series. The Kendall harmony coefficient is used to measure the ReHo value. By calculating the time series consistency (KCC value) between each voxel in the brain and its adjacent 26 voxels, the ReHo diagram of the whole brain of each subject can be obtained [6]. Then, the whole brain is averaged; that is, the ReHo value of each voxel is divided by the whole brain ReHo mean to achieve standardization. In order to further reduce noise and improve signal-to-noise ratio, Gaussian smoothing kernel with half height and width of 6 mm is used for spatial smoothing. The ReHo values of the two sets of subjects were statistically analyzed by paired *t*-test to obtain the different brain regions before and after acupuncture. Gaussian random field theory (GRF) is used for multiple comparison correction.

## 3. Research Results

A total of 20 female healthy subjects were included in this study, and all completed fMRI scanning before and after acupuncture. Using the method of ReHo analysis to analyze the fMRI data, it was found that the ReHo values of the left precuneus lobe, left central posterior gyrus, calcarine, left lingual gyrus, and cerebellum induced by electroacupuncture at uterine point were significantly lower than those before acupuncture. After GRF correction (voxel *P* < 0.05, cluster *P* < 0.05), there was significant difference (see Table 1 and Figure 1 for details).

## 4. Discussion

Acupuncture and moxibustion are more and more recognized by the medical community, and the mechanism of acupuncture and moxibustion is also being explored. With the development of science and technology, fMRI is a new imaging method in recent years. It has the unique advantages of no radiation, no bone artifacts, and multiparameter imaging. It has become one of the hotspots of acupuncture research. The principle is mainly to observe the change characteristics of image signal intensity according to the change of blood oxygen level by calculating the ratio of oxygenated hemoglobin to deoxyhemoglobin and the change of relative concentration of deoxyhemoglobin, combined with the paramagnetic characteristics of deoxyhemoglobin [7].

ReHo is a method for measuring similarity or coherence in voxel analysis of the whole brain. This method has been used to explain the relationship between neurovascular coupling and task activation [8], as well as the functional regulation of cognitive changes in subjects in a resting state [8]. However, there are few studies on the changes of ReHo in brain region caused by acupuncture. In this study, we found that acupuncture at uterine point can inhibit the neural activities of the precuneus, cerebellum, talform sulcus, lingual gyrus, and posterior central gyrus. In a previous study, Lin et al. reported that the higher the ReHo value, the stronger the synchronization of local neuronal activities, which is a compensatory response to metabolic abnormalities and blood flow changes related to adverse clinical outcomes [9]. Their results suggest that the reduction of ReHo may have a protective effect. In this study, we found that electroacupuncture at uterine points can reduce ReHo values in brain regions such as the precuneus lobe in healthy subjects. However, whether electroacupuncture at uterine point has neuroprotective effect needs further study.

Precuneus is considered to be one of the important regions related to emotion, cognition, and memory and related to mental disorders. It participates in the distributed network of cortical and subcortical regions and integrates self-generation and external information [10]. The precuneus can produce significant neural changes to inconsistent stimulation information [11]. The nerves distributed at uterine points have the same part as the ganglion segments of female reproductive organs such as the uterus, and studies have proved that acupuncture can cause changes in sex hormones [12]. Therefore, we speculate that the reduction of ReHo in precuneus is related to sex hormone fluctuations and emotional changes. The regulatory effect and clinical efficacy of acupuncture and moxibustion also show that acupuncture and moxibustion can maintain internal balance. Therefore, we speculate that the potential mechanism of acupuncture at uterine points in the treatment of gynecological and reproductive diseases may be related to the neural activity of precuneus, regulate the changes of female emotion, and restore the normal level of hormone.

As we all know, the basic function of the cerebellum is to maintain postural balance and coordinate random movement. Studies have also shown that the cerebellum plays a potential role in many functions such as cognition and emotion [13]. The literature suggests that [14] the cerebellum has a wide impact on the emotion, pain, and other negative emotions of female patients with premenstrual anxiety. Some scholars have found that [15], in patients with premenstrual syndrome, bilateral cerebellar falff decreases, and acupuncture at Sanyinjiao can induce bilateral cerebellar falff to increase. This study also proves that electroacupuncture at bilateral uterine points can affect the ReHo value of the cerebellum. Therefore, we believe that acupuncture at uterine points can regulate the activity of the cerebellum and then affect the changes of women's emotion and cognition.

The posterior central gyrus belongs to the parietal lobe, also known as the somatosensory center, and is part of the pain matrix. It may play a key role in regulating pain perception, including pain localization and pain intensity recognition. Ke et al. [16] reported that ReHo increased due to adaptive neuronal changes caused by long-term pain stimulation and biological response. Electroacupuncture at bilateral uterine points can reduce the ReHo value of the posterior central gyrus. We speculate that electroacupuncture at bilateral uterine points can affect the pain regulation function of the posterior central gyrus to a certain extent, which may be the effective mechanism of acupuncture at uterine points in the treatment of dysmenorrhea.

The calcarine sulcus and lingual gyrus are located in the visual cortex and play an important role in vision [17]. In addition, the study of Rehbein et al. [17, 18] also proved that, at the neural level, the increase of estradiol level was related to the decreased activation of the right lingual gyrus and left calcarine sulcus. In the present study, visual structures were involved in electroacupuncture at uterus points, suggesting that uterus points may be related to the treatment of visual impairment. Therefore, we speculated that electroacupuncture of bilateral uterine acupoints interferes with the changes of talus sulcus and lingual gyrus, thus improving the level of estradiol, which may be the neuroimaging mechanism of uterine acupoints for the treatment of reproductive diseases.

In conclusion, electroacupuncture at bilateral uterine points can affect the neural activities of brain areas such as the precuneus lobe, cerebellum, posterior central gyrus, talform sulcus, and lingual gyrus, which may be related to the fact that acupuncture at uterine points can regulate the level of reproductive hormone, emotional changes, and somatic sensation, so as to clarify the neural mechanism of acupuncture at Zigong point in the treatment of reproductive and gynecological diseases to a certain extent. However, further experiments are needed to prove whether this is related and consistent with the brain effect of acupuncture at uterine points under pathological conditions. In addition, the sample size of this study is too small, and only 20 volunteers were recruited. Although the number of participants is no less than that in previous similar studies [19–21], we believe that the number of volunteers in fMRI research is more than 20, which may obtain more convincing evidence. These problems will be solved in our future research.

## Figures and Tables

**Figure 1:** Different brain regions before and after acupuncture intervention.

**Table 1:** Different brain regions before and after acupuncture intervention.

Brain region	Hemisphere	Condition	MNI			Cluster size	Peak *t*
			*X*	*Y*	*Z*		
Precuneus	Left	After acupuncture < before acupuncture	-27	-66	48	456	-5.3196
Posterior gyrus							
Calcarine	Bilateral	After acupuncture < before acupuncture	0	-93	0	327	-5.7168
Lingual gyrus	Left						
Cerebellum	Bilateral	After acupuncture < before acupuncture	-6	-72	-18	357	-5.4967

MNI: Montreal Neurological Institute, Montreal Institute. The cluster of precuneus also includes functional brain areas such as the central posterior gyrus and superior parietal lobule. The cluster of the talform sulcus also includes functional brain regions such as the lingual gyrus, middle occipital gyrus, and inferior occipital gyrus.

## Data Availability

The datasets are available at http://www.oasis-brains.org/.
